# Calculation Model of Regional Economic Growth Efficiency by Intelligently Optimized Interunit Layout

This article has been retracted.

**DOI:** 10.1155/2022/9775900

**Published:** 2022-08-23

**Authors:** Xiufeng Song, Jingying Ke, Huayan Shen

**Affiliations:** ^1^School of Economics and Management, Nanchang Normal College of Applied Technology, Nanchang 330000, Jiangxi, China; ^2^Business School, Xiamen Institute of Technology, Xiamen 361000, Fujian, China; ^3^School of Economics and Management, Guangzhou City Construction College, Guangzhou 510925, China

## Abstract

With the development of the economy, especially since the reform and opening up, the actual conditions that China's economic development faces have also changed, and the development goals have also been adjusted accordingly. However, since the reform and opening up, China's economy has still largely relied on the extended reproduction of the extension type. It basically develops along a high-input, low-efficiency path. The effectiveness of regional economic development has always been one of the most important debates in economics, and it has attracted great attention in different countries and regions around the world. So far, people have conducted a lot of theoretical and practical research on the effectiveness of regional development and put forward many practical countermeasures. However, it has achieved little in practice, and the original form of high growth and low efficiency has not been effectively reversed. In this paper, economic development is divided into two parts. The first part consists of the impact of changes in the quantity of factors of production on economic growth and the impact of the efficiency of economic growth on the entire economy. The second part consists of the annual average efficiency of economic growth. The average annual contribution of various production factors to economic growth and the economic growth efficiency of changes in the allocation of capital industries were 6.21%, 5.02%, 4.05%, 3.9%, and 3.3%, respectively in the past five years.

## 1. Introduction

Economic growth has always been a hot topic in economic research. In the past, under the condition of low economic aggregate, low capital cost, and low pressure on resources and environment, strong input growth can still maintain a high growth rate. It accumulates wealth for society, and people's lives continue to improve. While people's material and cultural living standards continue to improve, people's needs continue to diversify, especially when the pressure on resources and the environment continues to increase, and the efficiency of economic development has been neglected. The speed of rapid economic growth based on input growth is constrained by many factors.

It is becoming clear that a number of factors are at play in the slowdown in regional economic growth. An effective way to reverse this situation is to reduce the dependence on increased investment and improve the efficiency of regional economic development. To this end, it is necessary to scientifically measure and evaluate the effect of economic development over a period of time, so as to promote the stable, rapid, and sustainable growth of the regional economy under the constraints of limited resources and environment.

The innovation of this paper is to examine the regional economic system from the perspective of system science and engineering. This paper systematically analyzes the various basic factors and their structure, function, and interaction. Through decomposition and synthesis, this paper finally summarizes them into five basic factors (increase in the quantity of labor input, growth in industrial capital per capita, change in the allocation of labor between industries, change in the allocation of capital between industries, and change in the ratio of industrial output to capital). This paper incorporates them into a relatively complete theoretical-empirical analysis framework to study their role in economic growth.

## 2. Related Work

Regarding regional economic growth, relevant scientists have conducted the following research. Wei Ren used an integrated perspective combined with a margin approach to weigh the impact of the strategy on the historical impact on economic growth and prosocial development in Northeast China. The results of the study show that the proposed strategy markedly increased regional economic growth and per capita income, increasing China's GDP and per capita GDP by 25.70% and 46.00%, respectively. The next phase of the strategy should emphasize increasing R&D and human capital investment on the basis of urban heterogeneity to prevent conservative path dependence and targeting of backward technologies [1]. Yongshi and Mingxing aimed to carry out an actual study on the correlation between the distribution industry and regional economic growth in Fujian Province. The findings show that the circulation industry is positively correlated with regional economic growth and that the circulation industry is an important cause of economic growth in the region. His had further researched the power system of the circulation industry for regional economic development, which showed that the distribution industry has a linkage effect, diffusion effect, and spillover effect on regional economic growth. Therefore, it is the leading and basic industry of the regional economy [2]. Chen examined the influence of foreign direct income in China on the growth of its economy. He used a panel dataset at the provincial level and employed regression techniques with fixed effects and instrumental variables. His found that both provincial-level OFDI and SOE OFDI have a positive impact on China's provincial-level economic growth. The positive impact of OFDI on provincial economic growth may be due to the reverse knowledge spillover of OFDI to the home province economy through demonstration and imitation, labor mobility, and backward and forward linkages of industries. Thus, it improved the productivity and efficiency of firms in the home province and contributed to the economic growth of the home province [3]. On the basis of the convergence theory, Mei first developed a convergence model for the difference in GDP per capita between less developed, developing, and developed regions. Then, he constructed a convergence model for the difference between energy intensity and GDP per capita. It was discovered that the growth of GDP average capita in China showed a tendency to converge, while the growth rate of energy intensity was a bit lower than the growth rate of GDP average capita. It is recommended that local governments should fully take into account the convergence characteristics of regional energy consumption differences when implementing energy conservation and emission reduction strategies. Both economic growth and energy conservation and emission reduction should be ensured to ensure sustainable economic growth [4]. Qiu et al. proposed a meta-heuristic scheduler intelligent ant colony optimization task offloading algorithm to offload IoT sensor application tasks in foggy environments. The results of the algorithm he presented were compared with the throttling scheduling algorithm and two biologically inspired algorithms such as modified particle swarm optimization and bee life algorithm. Numerical results show that in task offloading for IoT sensor applications, His proposed intelligent ant colony optimization algorithm that has a significant improvement in latency compared with throttling, MPSO, and BLA [5]. Melhem et al. presented a linear programming model for mixed integers. He optimized an integrative smart residential energy production and consumption system for renewable energy sources, storage systems with batteries, and connected vehicles to the grid. He proposed a heuristic technique to solve the problem of managing residential energy and minimizing the cost of electricity to the consumer. The result was to find a globally optimal solution for multiple consecutive days, substantially reducing the implementation time and delivering remarkable energy cost savings in the considered case [6]. Khan and Singh presented a comparative analysis of different performance metrics using standard benchmark functions and addressed the minimization of operating costs for smart microgrids. He modeled the proposed SMG. These include utility-connected power sources such as wind turbines, photovoltaics, fuel cells, microturbines, battery storage, electric vehicle technology, and diesel generators. He concluded with a detailed review of microgrid operating cost minimization techniques based on exhaustive investigation and implementation [7]. The studies provide a detailed analysis of regional economic growth and the application of intelligent optimization. It is undeniable that these studies have greatly promoted the development of the corresponding fields. We can learn a lot from methodology and data analysis. However, there are relatively few studies on intelligent optimization for regional economic growth, and it is necessary to fully apply these algorithms to research in this field.

## 3. Methods of Regional Economic Growth Efficiency Measurement Model

### 3.1. Intelligent Optimization

Smart optimization is an intelligent and automated scenario-based account optimization system. This article uses the platform's various optimization packages to easily and effectively improve promotion. Modeling technology plays a very important role in modern industrial production management and optimization. As production plants become larger and more complex, time-varying objects, nonlinearities, long delays, strong coupling, and other issues undermine modeling efforts. Modeling is becoming increasingly complex, leading researchers and engineers to constantly seek and discover new modeling techniques. The modeling methods can generally be divided into mechanical modeling, empirical modeling, and inverse formula modeling [8]. The general structure of empirical modeling is shown in Figure 1. Modeling is based on a large number of observed sample data of the process, and the input variables and prediction objects of the model are selected in this paper. The mathematical model is obtained through statistical analysis, data processing, or artificial intelligence, which is the system identification of nonlinear objects. The main content includes three tasks: acquisition and processing of process data, model selection, and model validation. Since the modeling process does not require the guidance of the system's explicit mechanism, this method is often used for nonlinear system modeling where the internal mechanism of the system is not easy to grasp, or the object is highly time-varying. Commonly used empirical modeling methods are as follows: univariate and multivariate linear regressions. It is based on least squares estimation and linear and nonlinear regressions of principal components, maximum likelihood system identification methods, etc.

Mechanism modeling is to establish the mathematical model of the object according to the actual system mechanism and according to the corresponding theory (such as mass conservation and dynamics, etc.) under certain assumptions. The mechanism model is easy to understand. The established model has a strong theoretical basis and can more accurately express the relationship between variables. The modeling process does not require too much process data. Therefore, it is often used for modeling single operating units or simple nonlinear industrial processes. For the large-scale industrial modeling process or the control object whose internal mechanism is complex and difficult to be grasped by people, the mechanism modeling is very difficult. In addition, with the aging of the thermal power plant equipment or the change in the operating conditions of the steam turbine unit, the mechanism model established under a specific working condition cannot provide a good prediction effect for other variable working conditions. Therefore, conventional mechanism modeling methods are difficult to meet the needs of industrial development.

Directional modeling methods generally include three stages: data preparation, reverse modeling, and model validation [9]. The general flow of reverse modeling is shown in Figure 2. Reverse modeling is a modeling method relative to forward modeling methods such as mechanism modeling and empirical modeling. Its main idea is to change the output of the modeling system into a known quantity by means of actual measurement or calculation, and infer the cause from the result as a reverse modeling strategy. The reverse modeling technology does not make any assumptions about the specific structure of the modeling system or the modeling object, but is a modeling technology based on experimental data. Since reverse modeling techniques are based on real data on how the modeled object operates, errors introduced by assumptions, and simplifications to the system can be avoided. More importantly, the operational data include not only the actual environmental factors of the modeled object but also the health status of the modeled object. Therefore, the established model is more accurate. Reverse modeling regards the modeling system as a black box, and uses the actual operation data to avoid manpower and material resource consumption in experimental modeling and improve the modeling efficiency. Inverse modeling of multivariable, strongly coupled systems also avoids problems such as mechanism modeling that is difficult to solve. Therefore, inverse modeling techniques are suitable for modeling complex thermal systems operating under multiple operating conditions, such as steam turbines.

Statistics-based machine learning technology is different from the asymptotic theory of traditional statistical research, which studies the limit characteristics when the number of samples tends to infinity. The former is an incomplete induction method. By training and learning a given limited sample, and inducting the dependency between the input sample and the output sample, it is expected that this relationship can be used to predict the unknown output more accurately. In practical engineering projects, the number of learning samples is often limited. This also makes it difficult for a traditional asymptotic theory to generalize the relationship between system input and output [10].

The purpose of SVM is not to accurately describe known samples but to minimize structural risk to improve making predictions about future samples as accurate as possible. The closer the prediction result is to the real output of the sample, it will not only lead to the infinite learning of the sample by the learning machine and the overlearning situation, but also meet the needs of the learning machine for the promotion ability under the limited sample [11]. The prediction process of SVM for finite samples is a solution process of a convex quadratic programming problem, which is compared with the local optimal solution obtained by the artificial neural network based on empirical risk minimization [12]. For nonlinear regression problems, SVM employs a kernel function to project nonlinear samples into a high-dimensional feature space to solve the problem, and the kernel skill subtly overcomes the curse of feature space dimensionality. SVM shows many unique advantages, such as it can avoid the curse of dimensionality and local minima, and has a strong generalization ability. Although SVM has many advantages described, it has also been widely used in practical engineering. However, it still has some challenges to deal with. For example, how to choose the most reasonable kernel function for different engineering problems; after the kernel function is determined, how to choose the parameters of the kernel function and the parameters of the SVM to ensure that the SVM has the best fitting ability and generalization ability; and how to use SVM to solve multiobjective regression problems more efficiently, these are the challenges that need to be faced [13].

(1) $$\begin{array}{c} C_{i\;d}^{k+1}=qC_{i\;d}^{k+1}+p_{1}r_{1}\left(L_{i\;d}^{k}-M_{i\;d}^{k}\right)+p_{2}r_{2}\left(L_{i\;d}^{k}-M_{i\;d}^{k}\right), \end{array}$$

(2) $$\begin{array}{c} M_{i\;d}^{k+1}=M_{i\;d}^{k}+C_{i\;d}^{k+1}, \end{array}$$

(3) $$\begin{array}{c} L_{u}=\frac{f_{u}}{\sum_{u=1}^{n}f_{u}}. \end{array}$$

*C*_*i*  *d*_^*k*^ is the speed of the particles, *L*_*i*  *d*_^*k*^ is the individual best position, *L*_*i*  *d*_^*k*+1^ is the global best position, *M*_*i*  *d*_^*k*^ is the current particle position, *k* is the current iteration count, and *q* is the inertia weight for initial velocity.

(4) $$\begin{array}{c} F_{T}\left(M_{a}\Rightarrow m_{b}\right)=\left\{\begin{array}{c} 1,f\left(m_{b}\right)\leq f\left(m_{a}\right),\\ e^{df/T},f\left(m_{b}\right)>f\left(m_{a}\right), \end{array}\right.. \end{array}$$

(5) $$\begin{array}{c} M=I_{1}+\left(\sum_{u=1}^{k}y_{u}\cdot 2^{u-1}\right)\cdot \frac{I_{2}-I_{1}}{2^{k}-1}. \end{array}$$

*f* is the fitness function.

(6) $$\begin{array}{c} q_{u}^{k}=\frac{1}{1+e^{\left|\gamma +\mu_{u}^{k-1}\left(k-1\right)\right|}}, \end{array}$$

(7) $$\begin{array}{c} \gamma =\ln\frac{1-q\max}{q\max}, \end{array}$$

(8) $$\begin{array}{c} \mu =\frac{q\max-q\min}{q\max}, \end{array}$$

*q* is the inertia weight, *k* is the current number of iterations of the algorithm, and *k*max is the maximum number of iterations of the algorithm.

(9) $$\begin{array}{c} k=\frac{2}{\left|2-\varpi -\sqrt{\varpi^{2}-4\omega }\right|}, \end{array}$$

*κ* is the contraction factor.

(10) $$\begin{array}{c} C_{i\;d}^{k+1}=\kappa \left(qC_{i\;d}^{k}+p_{1}r_{1}\left(L_{i\;d}^{k}-M_{i\;d}^{k}\right)+p_{2}r_{2}\left(L_{i\;d}^{k}-M_{i\;d}^{k}\right)\right), \end{array}$$

(11) $$\begin{array}{c} M_{i\;d}^{k+1}=M_{i\;d}^{k}+C_{i\;d}^{k+1}. \end{array}$$

*C*_*i*  *d*_^*k*^ is the speed of the particles and *L*_*i*  *d*_^*k*^ is the individual best position.

(12) $$\begin{array}{c} {\left[a\left(m_{1},f_{1}\left(m\right)\right),a\left(m_{2},f_{2}\left(m\right)\right),\ldots a\left(m_{b},f_{b}\left(m\right)\right)\right]}^{T}=0, \end{array}$$

(13) $$\begin{array}{c} \underset{1\leq u\leq b}{\min}\left\{m_{u},f_{u}\left(m\right)\right\}=0,u=1,2,\ldots ,n, \end{array}$$

$\underset{1\leq u\leq b}{\min}\left\{m_{u},f_{u}\left(m\right)\right\}$ is the minimal form.

(14) $$\begin{array}{c} A\left(m,\eta \right)=\left[\begin{array}{c} m_{1}+f_{1}\left(m\right)-\sqrt{{\left(m_{1}-f_{1}\left(m\right)\right)}^{2}+\eta }\\ \vdots \\ m_{b}+f_{b}\left(m\right)-\sqrt{{\left(m_{b}-f_{b}\left(m\right)\right)}^{2}+\eta } \end{array}\right], \end{array}$$

(15) $$\begin{array}{c} F_{l}\left(m\right)=\frac{1}{l}\ln\left\{\sum_{u=1}^{b}\exp\left[lf_{1}\left(m\right)\right]\right\}. \end{array}$$

*F*_*l*_(*m*). is the agglomeration function.

(16) $$\begin{array}{c} f\left(m\right)=\underset{1\leq u\leq b}{\max}\left\{\left|f_{u}\left(m\right)\right|\right\}, \end{array}$$

(17) $$\begin{array}{c} \underset{1\leq u\leq b}{\min}\left\{m_{u},f_{u}\left(m\right)\right\}=-\max\left\{-m_{u},-f_{u}\left(m\right)\right\}, \end{array}$$

*f*(*m*) is the nonsmooth function.

The nonlinear complementarity problem approximates a smooth system of formulas as follows:

(18) $$\begin{array}{c} {\left[a_{\omega }\left(m_{1},f_{1}\left(m\right)\right),a_{\omega }\left(m_{2},f_{2}\left(m\right)\right),\ldots ,a_{\omega }\left(m_{b},f_{b}\left(m\right)\right)\right]}^{t}=0, \end{array}$$

(19) $$\begin{array}{c} a_{\omega }\left\{m_{u},f_{u}\left(m\right)\right\}=-\omega \left\{\exp\left(-m_{u}/\omega \right)+\exp\left(-f_{u}\left(m\right)/\omega \right)\right\}, \end{array}$$

(20) $$\begin{array}{c} F\left(m\right)=\left[\begin{array}{c} \frac{2}{5}m_{1}^{3}+m_{1}m_{2}+\frac{1}{2}m_{2}\\ m_{1}^{2}+m_{2}^{2}-\frac{1}{2} \end{array}\right], \end{array}$$

*a*_*ω*_{*m*_*u*_, *f*_*u*_(*m*)}. is the approximate smooth function and *F*(*m*) is the nonlinear complementary problems.

At present, the commonly used modeling methods include the neural network modeling method, extreme learning machine modeling method, support-vector machine modeling, and other methods. Model verification is the key link of the reverse modeling method. The correctness of the model is ensured by verifying the modeling accuracy, and then, the model is modified according to the model differences, and the appropriate model parameters are selected to obtain the final model that meets the requirements.

Model validation is one of the indispensable steps in reverse modeling. The commonly used method is as follows: it divides the modeling data into two parts; one part is used to train the model, and the other part is used to validate the model. It inputs the data used to verify the model into the trained model to obtain the corresponding predicted output value and compares the target value of the verification model data with the predicted output value. If the error index meets the engineering requirements, it can be considered that the model is correct.

### 3.2. Regional Economic Growth Efficiency

Areas can be divided into two categories: natural areas and socioeconomic areas. The macroscopic and dynamic research on economic policies and conditions of population, environment, and capital formation in the region lays the foundation of regional economic theory. From the division of administrative divisions, we can intuitively see the degree of unbalanced economic development between regions and the gap between various economic indicators [14].

Regional economic growth refers to the economic benefits created by the action of certain material/materials and human capital in the production field within a certain spatial range divided by administrative regions. The reason why we study regional economic growth here is that understanding the influencing factors and ways of causing differences in economic growth between regions is beneficial to the establishment of differential policies. Especially under the current economic development environment, there are obvious gradient differences in the level of economic development, and a correct understanding of the regional economy can narrow the differences in regional economic development as soon as possible [15]. Regional economic growth specifically refers to the degree to which the provincial resident residents use local material materials and labor to improve their economic level within a certain period of time under the same technical level. Regional economic growth is regional, differentiated, integrated, and related.

In the existing research results, the measurement of economic growth efficiency is generally achieved through the following methods: first, the economic efficiency in different periods is measured, and then, the change in economic efficiency is compared with the change in output or input. Therefore, the measurement method of “economic efficiency” in these studies also becomes the basis for measuring “economic growth efficiency.”

*Traditional Index Method*. The advantage of this type of measurement method is that the principle is simple. It only uses elementary mathematics knowledge, and the calculation is convenient. However, when calculating the output quantity index and the input quantity index, it is necessary to fix the corresponding prices in the same period if the Laplace quantity index is used for calculation. They are all fixed at the base period. If the Paasche quantity index is used, it is fixed at the reporting period, which means it is assumed that outputs have the same price in the base and reporting periods, and inputs have the same prices in the base and reporting periods. This is clearly inconsistent with reality. In the case of large price changes in the base period and the reporting period, this method cannot reasonably reflect the economic efficiency.

Based on the new economic geography theory based on economies of scale, externalities, and agglomeration economies, this paper analyzes the dynamics and mechanisms of regional economic disparities. The typical representative of this theory is Krugman, who explained the relationship between the geographical selection of manufacturing enterprises and changes in market demand through a simple model [16]. The geographic agglomeration of industries supported by decreasing costs has resulted in continued regional economic growth and continued productivity gains. When the utility of economic agglomeration occurs, the area where it initially won a competitive advantage is more agglomerated. Due to the existence of market mechanisms, the continuous accumulation of material materials and labor in the region has led to the widening of differences between regions.

The regional convergence and divergence theory is based on the new geographic economic model. This paper studies the convergence and divergence of regional income. Convergence generally occurs only in wealthy areas, and divergence is more likely to occur in areas with poor economic conditions. Trade liberalization has led to a long-term trend of regional convergence and divergence, and industrial structure and spatial distance have played an important role [17]. This article provides the basic basis for understanding the trends, characteristics, and causes of regional convergence and divergence, and for narrowing the gap between regions and realizing regional integration.

The description object of efficiency is a process. In the first interpretation, efficiency is used to describe the process of a job. In the second explanation, it is used to describe the process of mechanical and electrical work. In practical applications, efficiency can be used to describe various processes; for example, production efficiency can be used to describe the production process. The learning process can be described by learning efficiency; the public management work process can be described by administrative efficiency; and the photoelectric conversion process in natural science can be described by the conversion efficiency of light and electricity and others [18].

Efficiency is the result of comparing the effect with the elements that produce the effect. Efficiency is the result of comparing the amount of work done and the time invested, that is, the amount of work done per unit time. Efficiency is the result of the comparison between useful work and total work input [19]. The two explanations of efficiency can be combined into a general concept. Efficiency is one of the indicators to evaluate the operating state of a process, and it is the result of comparing the effect with the elements that produce the effect. If both the effect and the input can be measured by quantitative indicators and compared by the method of ratio, then it can be said that efficiency is the ratio of effect to the factor that produces the effect, that is, the effect produced by one unit of factor [20].  Figure 3 shows the relationship between energy efficiency and regional economic growth efficiency.

It refers to output per capita as labor productivity and studies it as the efficiency of labor input. Accordingly, the specific definition of economic growth as economic growth refers to the continuous growth of the total output during the operation of the economic system of a country or region. The regional economic system not only has the general characteristics of the economic system but also has its particularity in the specific performance. There is a part-to-whole relationship between the various economic elements in the system and the regional economic system [21]. Each economic element is in a subordinate position in the regional economic system, and its function must be adapted to the overall regional economy. However, this kind of integrity is based on the perspective of economic regions, not the whole of the national economic system, nor the whole of a certain industry or a certain microeconomic system. The hierarchy of the economic system refers to the hierarchical order of the constituent elements of the economic system in terms of status, role, structure, and function. For a regional economic system, it is a system relative to its internal subsystems, and it is a subsystem of the macroeconomic system [22].

An open system is a system that exists to exchange matter, energy, and information with the external environment. Almost all natural systems are open systems. Systems that are completely isolated from the outside world do not actually exist. A very open system means that it exchanges matter, energy, and information with the environment on a large scale and in many different ways [23]. In contrast, the openness of China's regional economic system is manifested in that it is constrained by the natural environment, such as China's natural resources, ecological environment, and resource abundance. It is also constrained by the socioeconomic environment, such as macroeconomic systems, economic institutions, and demographic conditions. At the same time, it is also closely related to other external regional economic systems. In general, economic systems are more complex than engineering systems. However, regional economic systems are generally simpler than macroeconomic systems but more complex than microeconomic systems. As shown in Figure 4, there is a nonlinear relationship between regional economic growth and energy efficiency and the flow of production factors.

The main body of the economic system is the people. Due to the differences in people's thinking, judgment, decision-making, and preferences, the economic system with participation has obvious characteristics such as uncertainty and ambiguity. Compared with the macroeconomic system, due to the relatively small scale of the regional economic system, human decision-making may produce effects more quickly, so its uncertainty is more obvious [24]. The goals of the economic system may involve economic benefits, social benefits, and ecological and environmental goals. Sometimes it has to consider both long-term goals and short-term goals, and so on. The regional economic system also has a variety of goals, but some of them are consistent with the macro- or microeconomic system, and some may be contradictory. Compared with other economic systems, a specific regional economic system often has its own specific internal conditions and external macroenvironment. It may also enjoy special economic policies, have special decision-makers with specific abilities or preferences, and so on. It thus forms the characteristics that distinguish it from the macroeconomic system and other regional economic systems [25].

## 4. Experiments on the Calculation Model of Regional Economic Growth Efficiency

The differential evolution algorithm is an optimization algorithm based on population intelligence theory. The intelligence of the population is generated by the cooperation and competition among the individuals within the population, which guides the optimization search. Compared with the evolutionary algorithm, the differential evolution algorithm adopts a search strategy based on the global population. It adopts real-number coding, simple difference-based transformation operation, and single-competition survival strategy, which reduce the complexity of genetic operation. At the same time, the unique memory capability of the differential evolution algorithm enables it to dynamically monitor the current search state. It adjusts the search strategy in a globally highly convergent and robust manner without any problem feature information. This is suitable for solving some optimization problems in complex environments that cannot be solved by traditional mathematical design methods. As shown in Figure 5, it is the flowchart of the standard differential evolution algorithm for the layout of intelligent optimization in cells.

The common genetic algorithm and particle swarm algorithm are used for calculation, and the optimal value, fitness value, mean square error, and calculation time are listed.  Table 1 shows the verification results.

The simulated annealing genetic algorithm and the improved particle swarm algorithm are used for calculation, and the verification results are shown in Table 2.

Applying the intelligent optimization algorithm to solve the complementary problem gets rid of the trouble of selecting the initial point, and the value obtained by the algorithm is closer to the optimal value of the complementary problem. The verification results are shown in Tables 3 and 4.

Economic growth efficiency is an index that measures the effect of changes in efficiency factors on economic growth during the operation of the economic system. It is equal to the remaining effect after removing the effect of changes in the quantity of factor inputs in economic growth. Assuming that the number of input factors is constant, if the economic growth efficiency is higher, the economic growth will be faster.  Figure 6 shows the calculation process of the regional economic growth efficiency.

Since the reform and opening up, a province's economy has also experienced rapid growth, but its economic growth process is similar to that of the whole country, featuring high investment, high consumption, and low efficiency.  Figure 7 shows the economic growth rate and industrial growth rate of a province over the years. It can be seen that since the reform and opening up, Hebei's economic growth has fluctuated quite a lot, and it has basically gone through two stages with obvious characteristics. The economy has entered a relatively stable high-speed growth stage, and the volatility of economic growth has gradually weakened. Overall, the province's economy has achieved rapid growth since the reform and opening up.

Figure 8 shows the current price of the nominal output and the three industrial added-value indices. It can be seen that using the GDP index and formula (1) to calculate the actual GDP should be equal to the sum of the actual added value of each industry, but the actual calculation found that there is a certain gap between them. This should be caused by the different accounting methods and accounting calibers of the added-value index and regional GDP index of various industries.

The fixed capital stock is shown in Figure 9. This paper studies the relationship between the total fixed capital formation of various industries in the province and the fixed-asset investment of the corresponding industry, and finds that there is a very significant linear correlation between them.

As shown in Figure 10, the output of each industry, the proportion of output, the growth rate of labor force, and the growth rate of the regional economy are still higher than the annual average. However, the growth rates of regional GDP and value added of individual industries generally declined. This suggests that the region has already shown the first signs of an economic slowdown in recent years, which could lead to further declines if no countermeasures are taken.

An economic region is an economic and social cluster resulting from human economic activity. It exists objectively around the economic center, and it has specific spatial components and cannot be arbitrarily subdivided. The establishment and strict enforcement of a system for the protection of land, water, and other natural resources will reduce the waste of water and land resources and provide a basis for the development of modern agriculture, forestry, animal husbandry, and fisheries. It improves the equipment level of modern agriculture, forestry, animal husbandry, and fishery. It utilizes advanced production equipment and tools to strengthen basic industries. At the same time, it accelerates the technological innovation of agriculture, forestry, animal husbandry, and fishery. It strengthens closely related scientific and technological research and development. It strongly encourages the promotion and application of biotechnology and information technology. It promotes the transformation of scientific and technological achievements into practical productivity, and improves the scientific and technological content of research and development of agriculture, forestry, animal husbandry, and fishery.

## 5. Discussion

The market allocation mechanism of human capital is not perfect. The human resource market generally not only realizes the primary function of a negotiation place, but does not realize the important function of adjusting the supply and demand relationship by using market laws. Intermediary services in the middle and senior talent market are basically monopolized by government-affiliated agencies, which lack the motivation to compete and improve service levels. Institutional innovation is not enough, and the guarantee capacity for improving efficiency is weak. This is mainly reflected in the insufficient application of national macroeconomic policies. At present, China's regional economic development policy is conducive to the economic development of this province. However, in order to make full use of the national macroeconomic policy orientation, unify the national macropolicy objectives and the institutional innovation objectives of Hebei Province to promote institutional innovation in the province, and improve the level and success rate of institutional innovation, the province needs to further think and plan. Based on the lack of institutional supply in cross-regional economic cooperation, the role of the government in institutional innovation is inaccurate. At present, institutional innovation in the province relies too much on government behavior, and the degree of business participation is not high. During the implementation of some new policies, the phenomenon of government departments is single-handedly appeared, resulting in the inefficiency of institutional innovation in the implementation process.

In terms of efficiency factors, changes in the division of labor among industries are basically in line with the laws of the economy. They tend to favor economic growth because they are a significant source of efficiency gains. Changes in the capital index of industrial production have little effect on growth and growth efficiency. In the long run, changes in the allocation of capital across industries have a negative impact on growth and growth efficiency. The analysis of the evolution of profitability factors at the sectoral level shows that the flow of labor among industries is relatively flexible and basically in line with economic laws. The changes in the allocation of capital among industries have been unreasonable for a long time. It is mainly reflected in the primary and secondary industries. However, in recent years, the output-capital ratio of the tertiary industry is too low and has been declining for a long time. This is an important reason for the low contribution of the industrial output-capital ratio of the province to economic growth, and in recent years, it has deteriorated to the extent that it has seriously hindered economic growth.

## 6. Conclusions

Regional competitiveness refers to the ability of a region to attract and compete for resources, and the ability to optimize and rationally allocate resources to achieve sustainable, comprehensive, and coordinated development and sustainable regional competitive advantage. The strength of regional competitiveness directly affects the strength of a region's economic development. If we continue to rely on massive investment to drive rapid economic growth while ignoring the value of capital and the rational allocation of resources, and the need to acquire basic and critical technologies as soon as possible, it will inevitably lead to a scarcity of resources. It further increases environmental pressures, undermines the region's ability to attract investment, reduces self-sustaining innovation, and ultimately undermines regional competitiveness, growth, and employment. This paper introduces the intelligent optimized interunit layout to study the regional economic growth efficiency. In this paper, the preliminary prediction research is carried out. In view of the limited data sources and academic level, there are inevitably some omissions in the research. The analysis of the status quo analysis stage is not thorough enough, and it only shows the changes in relevant indicators and lacks internal judgment analysis. At the stage of theoretical research, this paper does not have a deep grasp of the theory. The measurement model can only give the measurement method of the regional economic growth efficiency. How to combine it with various macroeconomic and microeconomic factors that affect the efficiency of regional economic growth and incorporate it into the analytical framework of economic growth efficiency needs to be further studied.

## Figures and Tables

**Figure 1:** Empirical modeling general structure.

**Figure 2:** General flow of reverse modeling.

**Figure 3:** The relationship between energy efficiency and regional economic growth efficiency.

**Figure 4:** Nonlinear relationship.

**Figure 5:** Standard differential evolution algorithm flowchart.

**Figure 6:** Regional economic growth efficiency calculation process.

**Figure 7:** Economic growth rate and industrial growth rate over the years.

**Figure 8:** Current price of the nominal output and three industrial added-value indices.

**Figure 9:** Fixed capital stock.

**Figure 10:** Labor force growth rate.

**Table 1:** Algorithm verification results.

Initial point	Number of iterations	Iterative result	Time (s)
(0, 1)	5	(0,0,707208)	0.5
(1, 1)	8	(0,0,707307)	0.7
(10, 10)	15	(0,0,707307)	1.5
(−10, −10)	35	(0,855487,0)	3.4

**Table 2:** Validation results I.

Algorithm	The optimal value	Fitness value	Mean squared error	Time (s)
GA	(2.141e-06,0.707)	1.369e-05	2.1229e-14	95
PO	(9.076e-04,0.792)	1.067e-04	8.4319e-08	35
SA	(2.059e-10,0.716)	5.072e-14	8.1467e-15	190
Ic	(2.192e-02,0.771)	7.058e-18	9.0868e-35	42

**Table 3:** Validation results II.

Algorithm	The optimal value	Fitness value	Mean squared error	Time (s)
GA	(2.002, 0.314, 0.994, 0.0165)	0.8439	7.889e-05	104
PO	(2.078, 0.610, 0.924, 0.0707)	0.0362	0.015	52
SA	(2.008, 0.015, 0.931, 0.0142)	1.056e-08	5.718e-08	261
Ic	(2.000, 0.251, 0.705, 0.0562)	2.323e-15	0	57

**Table 4:** Validation results III.

Algorithm	The optimal value	Fitness value	Mean squared error	Time (s)
GA	(2.71e-05, 0.644, 0.244)	0.5049	8.3424e-05	108
PO	(5.34e-04, 0.757, 0.686)	0.2414	0.014	54
SA	(3.76e-06, 0.413, 0.534)	6.516e-05	3.3248e-05	298
Ic	(6.55e-08, 0.003, 0.312)	4.632e-12	8.5478e-12	87

## Data Availability

No data were used to support this study.
